# Diaqua­bis(pyridine-2-carboxyl­ato-κ^2^ *N*,*O*)cobalt(II)

**DOI:** 10.1107/S1600536808010507

**Published:** 2008-04-18

**Authors:** G. S. Huang

**Affiliations:** a College of Chemistry & Chemical Engineering, Provincial Key Laboratory of Coordination Chemistry, Jinggangshan University, Jian 343009, People’s Republic of China

## Abstract

In the mol­ecule of the title compound, [Co(C_6_H_4_NO_2_)_2_(H_2_O)_2_], the coordination environment around the Co^II^ atom is distorted octahedral; two N and two O atoms of the pyridine-2-carboxylate ligands lie in the equatorial plane and the two water O atoms in the axial positions. In the crystal structure, inter­molecular O—H⋯O hydrogen bonds link the mol­ecules, forming a supra­moleular network structure.

## Related literature

For general background, see: Desiraju (1997 ▶); Braga *et al.* (1998 ▶); McCann *et al.* (1996 ▶); Wai *et al.* (1990 ▶); Yaghi *et al.* (1996 ▶); Min & Lee (2002 ▶); Maira *et al.* (2001 ▶). For bond-length data, see: Allen *et al.* (1987 ▶).

## Experimental

### 

#### Crystal data

[Co(C_6_H_4_NO_2_)_2_(H_2_O)_2_]
*M* *_r_* = 339.17
Monoclinic,
*a* = 11.7401 (3) Å
*b* = 8.9994 (6) Å
*c* = 14.9211 (3) Å
β = 105.985 (2)°
*V* = 1515.52 (11) Å^3^
*Z* = 4
Mo *K*α radiation
μ = 1.16 mm^−1^
*T* = 273 (2) K
0.24 × 0.18 × 0.08 mm

#### Data collection

Bruker APEXII area-detector diffractometer
Absorption correction: multi-scan (*SADABS*; Sheldrick, 1996 ▶) *T*_min_ = 0.770, *T*_max_ = 0.918
9384 measured reflections
2926 independent reflections
2065 reflections with *I* > 2σ(*I*)
*R*_int_ = 0.042

#### Refinement

*R*[*F* ^2^ > 2σ(*F* ^2^)] = 0.060
*wR*(*F* ^2^) = 0.227
*S* = 1.07
2926 reflections
200 parameters
6 restraints
H atoms treated by a mixture of independent and constrained refinement
Δρ_max_ = 0.83 e Å^−3^
Δρ_min_ = −0.62 e Å^−3^

### 

Data collection: *APEX2* (Bruker, 2005 ▶); cell refinement: *SAINT* (Siemens, 1996 ▶); data reduction: *SAINT*; program(s) used to solve structure: *SHELXS97* (Sheldrick, 2008 ▶); program(s) used to refine structure: *SHELXL97* (Sheldrick, 2008 ▶); molecular graphics: *SHELXTL* (Sheldrick, 2008 ▶); software used to prepare material for publication: *SHELXTL*.

## Supplementary Material

Crystal structure: contains datablocks I, global. DOI: 10.1107/S1600536808010507/hk2450sup1.cif

Structure factors: contains datablocks I. DOI: 10.1107/S1600536808010507/hk2450Isup2.hkl

Additional supplementary materials:  crystallographic information; 3D view; checkCIF report

## Figures and Tables

**Table:** 

Co1—O1	2.150 (3)
Co1—O2	2.162 (3)
Co1—O3	2.151 (3)
Co1—O5	2.153 (3)
Co1—N1	2.284 (4)
Co1—N2	2.274 (3)

**Table:** 

O1—Co1—O2	84.68 (13)
O1—Co1—O3	167.36 (12)
O1—Co1—O5	98.78 (12)
O2—Co1—O3	92.63 (13)
O2—Co1—O5	95.35 (13)
O3—Co1—O5	93.75 (12)
O1—Co1—N1	86.44 (14)
O2—Co1—N1	163.96 (15)
O3—Co1—N1	98.83 (14)
O5—Co1—N1	72.84 (12)
O1—Co1—N2	93.86 (12)
O2—Co1—N2	98.99 (14)
O3—Co1—N2	74.33 (12)
O5—Co1—N2	161.68 (13)
N1—Co1—N2	94.91 (13)

**Table 2:** Hydrogen-bond geometry (Å, °)

*D*—H⋯*A*	*D*—H	H⋯*A*	*D*⋯*A*	*D*—H⋯*A*
O1—H1*B*⋯O4^i^	0.784 (18)	1.98 (3)	2.733 (4)	161 (4)
O1—H1*A*⋯O5^ii^	0.82	1.88	2.679 (4)	164
O2—H2*B*⋯O4^iii^	0.771 (16)	1.959 (16)	2.712 (4)	166 (3)
O2—H2*A*⋯O6^ii^	0.82	1.96	2.699 (5)	149

Symmetry codes: (i) ; (ii) ; (iii) .

## supplementary crystallographic information

### Comment

In the synthesis of crystal structures by design, the assembly of molecular units in predefined arrangements is a key goal (Desiraju, 1997; Braga *et al.*,  1998). Due to carboxyl groups are one of the most important classes of biological ligands, the coordination of metal-carboxyl groups complexes are of critical importance in biological systems, organic materials and coordination chemistry. Recently, carboxyl groups with variable coordination modes have been used to construct metal-organic supramolecular structures (McCann *et al.*,  1996; Wai *et al.*,  1990; Yaghi *et al.*, 1996; Min & Lee 2002; Maira *et al.*,  2001). We report herein the crystal structure of the title compound, (I).

In the molecule of (I) (Fig. 1), the ligand bond lengths  (Allen *et al.*, 1987) and angles are within normal ranges. The two N and the two O atoms of the two pyridine-2-carboxylato ligands in the equatorial plane around the Co^II^ atom form a distorted square-planar arrangement, while the  distorted octahedral coordination is completed by the two O atoms of water molecules in the axial positions (Table 1 and Fig. 1). The Co-O bonds [average 2.154 (3) Å] are somewhat shorter than the Co-N distances [average 2.279 (3) Å].

In the crystal structure, intermolecular O-H···O hydrogen bonds (Table 2) link the molecules to form a supramoleular network structure (Fig. 2), in which they may be effective in the stabilization of the structure.

### Experimental

The title compound was synthesized using hydrothermal method in a 23 ml Teflon-lined Parr bomb. Cobalt(II) chloride hexahydrate (47.6 mg, 0.2 mmol), pyridine-2-carboxylic acid (49.2 mg, 0.4 mmol) and distilled water (6 g) were placed into the bomb and sealed. The bomb was then heated under autogenous pressure up to 413 K over the course of 7 d and allowed to cool at room temperature for 24 h. Upon opening the bomb, a clear colorless solution was decanted from small pink crystals. These crystals were washed with distilled water followed by ethanol, and allowed to air-dry at room temperature.

### Refinement

H1B and H2B (for H_2_O) were located in difference syntheses and refined isotropically [O-H = 0.784 (18) and 0.771 (16) Å, U_iso_(H) = 0.065 (16) and 0.035 (12) Å^2^]. The remaining H1A and H2A (for H_2_O) and aromatic H atoms were positioned geometrically, with O-H = 0.82 Å (for H_2_O) and C-H = 0.93 Å for aromatic H, and constrained to ride on their parent atoms, with U_iso_(H) = xU_eq_(C,O), where x = 1.2 for aromatic H atoms and x = 1.5 for all other H atoms.

### Crystal data

**Table:**

[Co(C_6_H_4_NO_2_)_2_(H_2_O)_2_]	*F*_000_ = 692
*M**_r_* = 339.17	*D*_x_ = 1.486 Mg m^−^^3^
Monoclinic, *P*2_1_/*n*	Mo *K*α radiation λ = 0.71073 Å
Hall symbol: -P 2yn	Cell parameters from 2863 reflections
*a* = 11.7401 (3) Å	θ = 2.6–23.8º
*b* = 8.9994 (6) Å	µ = 1.16 mm^−^^1^
*c* = 14.9211 (3) Å	*T* = 273 (2) K
β = 105.985 (2)º	Plate, pink
*V* = 1515.52 (11) Å^3^	0.24 × 0.18 × 0.08 mm
*Z* = 4	

### Data collection

**Table:**

Bruker APEXII area-detector diffractometer	2926 independent reflections
Radiation source: fine-focus sealed tube	2065 reflections with *I* > 2σ(*I*)
Monochromator: graphite	*R*_int_ = 0.042
*T* = 273(2) K	θ_max_ = 26.0º
φ and ω scans	θ_min_ = 2.0º
Absorption correction: multi-scan(SADABS; Sheldrick, 1996)	*h* = −14→14
*T*_min_ = 0.770, *T*_max_ = 0.918	*k* = −11→11
9384 measured reflections	*l* = −18→17

### Refinement

**Table:**

Refinement on *F*^2^	Secondary atom site location: difference Fourier map
Least-squares matrix: full	Hydrogen site location: inferred from neighbouring sites
*R*[*F*^2^ > 2σ(*F*^2^)] = 0.060	H atoms treated by a mixture of independent and constrained refinement
*wR*(*F*^2^) = 0.227	*w* = 1/[σ^2^(*F*_o_^2^) + (0.152*P*)^2^ + 0.1958*P*] where *P* = (*F*_o_^2^ + 2*F*_c_^2^)/3
*S* = 1.07	(Δ/σ)_max_ < 0.001
2926 reflections	Δρ_max_ = 0.83 e Å^−^^3^
200 parameters	Δρ_min_ = −0.62 e Å^−^^3^
6 restraints	Extinction correction: none
Primary atom site location: structure-invariant direct methods	

### Special details

**Table:**

Geometry. All e.s.d.'s (except the e.s.d. in the dihedral angle between two l.s. planes) are estimated using the full covariance matrix. The cell e.s.d.'s are taken into account individually in the estimation of e.s.d.'s in distances, angles and torsion angles; correlations between e.s.d.'s in cell parameters are only used when they are defined by crystal symmetry. An approximate (isotropic) treatment of cell e.s.d.'s is used for estimating e.s.d.'s involving l.s. planes.
Refinement. Refinement of F^2^ against ALL reflections. The weighted R-factor wR and goodness of fit S are based on F^2^, conventional R-factors R are based on F, with F set to zero for negative F^2^. The threshold expression of F^2^ > 2sigma(F^2^) is used only for calculating R-factors(gt) etc. and is not relevant to the choice of reflections for refinement. R-factors based on F^2^ are statistically about twice as large as those based on F, and R- factors based on ALL data will be even larger.

### Fractional atomic coordinates and isotropic or equivalent isotropic displacement parameters (Å^2^)

**Table:**

	*x*	*y*	*z*	*U*_iso_*/*U*_eq_	
Co1	0.74558 (5)	0.85905 (7)	0.62775 (4)	0.0500 (3)	
O1	0.8193 (3)	0.7460 (4)	0.7578 (2)	0.0528 (8)	
H1A	0.7662	0.7036	0.7737	0.079*	
H1B	0.8854 (17)	0.719 (5)	0.773 (3)	0.065 (16)*	
O2	0.5921 (3)	0.8896 (4)	0.6792 (3)	0.0562 (9)	
H2A	0.5826	0.8156	0.7083	0.084*	
H2B	0.546 (3)	0.953 (3)	0.673 (3)	0.035 (12)*	
O3	0.6510 (3)	0.9270 (3)	0.48901 (19)	0.0497 (8)	
O4	0.5390 (3)	0.8577 (3)	0.3503 (2)	0.0560 (9)	
O5	0.8183 (3)	1.0767 (4)	0.6673 (2)	0.0512 (8)	
O6	0.9716 (3)	1.2287 (4)	0.6898 (3)	0.0724 (11)	
N1	0.9333 (3)	0.8598 (4)	0.6113 (3)	0.0504 (9)	
N2	0.6905 (3)	0.6452 (4)	0.5461 (2)	0.0406 (8)	
C1	0.6032 (3)	0.8310 (5)	0.4295 (3)	0.0423 (9)	
C2	0.6267 (3)	0.6693 (5)	0.4583 (3)	0.0392 (9)	
C3	0.5838 (4)	0.5535 (5)	0.3968 (3)	0.0533 (11)	
H3	0.5424	0.5722	0.3351	0.064*	
C4	0.6040 (4)	0.4115 (6)	0.4293 (3)	0.0552 (11)	
H4	0.5727	0.3319	0.3906	0.066*	
C5	0.6700 (4)	0.3862 (5)	0.5184 (4)	0.0552 (12)	
H5	0.6864	0.2897	0.5404	0.066*	
C6	0.7120 (4)	0.5054 (5)	0.5755 (3)	0.0495 (10)	
H6	0.7569	0.4880	0.6364	0.059*	
C7	0.9224 (4)	1.1095 (5)	0.6665 (3)	0.0513 (11)	
C8	0.9904 (4)	0.9869 (5)	0.6340 (3)	0.0489 (11)	
C9	1.1060 (4)	1.0058 (7)	0.6312 (4)	0.0704 (15)	
H9	1.1443	1.0961	0.6485	0.085*	
C10	1.1635 (6)	0.8917 (7)	0.6029 (6)	0.091 (2)	
H10	1.2403	0.9039	0.5983	0.109*	
C11	1.1064 (6)	0.7581 (8)	0.5811 (6)	0.102 (2)	
H11	1.1445	0.6768	0.5639	0.123*	
C12	0.9906 (5)	0.7476 (6)	0.5856 (5)	0.0772 (17)	
H12	0.9510	0.6578	0.5698	0.093*	

### Atomic displacement parameters (Å^2^)

**Table:**

	*U*^11^	*U*^22^	*U*^33^	*U*^12^	*U*^13^	*U*^23^
Co1	0.0509 (5)	0.0450 (5)	0.0472 (5)	−0.0007 (3)	0.0018 (3)	−0.0005 (2)
O1	0.0397 (16)	0.060 (2)	0.0502 (18)	0.0013 (15)	−0.0015 (13)	0.0150 (14)
O2	0.056 (2)	0.0450 (19)	0.070 (2)	0.0125 (16)	0.0209 (17)	0.0143 (16)
O3	0.0515 (17)	0.0412 (18)	0.0466 (17)	−0.0020 (13)	−0.0031 (13)	0.0045 (13)
O4	0.0550 (19)	0.052 (2)	0.0467 (18)	0.0079 (14)	−0.0106 (14)	0.0083 (13)
O5	0.0467 (17)	0.0448 (18)	0.0613 (19)	−0.0019 (14)	0.0135 (14)	−0.0096 (15)
O6	0.078 (2)	0.059 (2)	0.089 (3)	−0.0299 (19)	0.037 (2)	−0.031 (2)
N1	0.049 (2)	0.046 (2)	0.059 (2)	−0.0010 (17)	0.0189 (18)	−0.0046 (17)
N2	0.0418 (18)	0.037 (2)	0.0366 (18)	−0.0012 (14)	0.0011 (14)	0.0024 (13)
C1	0.0331 (19)	0.049 (2)	0.040 (2)	0.0023 (17)	0.0035 (16)	0.0025 (18)
C2	0.0334 (19)	0.041 (2)	0.039 (2)	−0.0012 (16)	0.0032 (15)	−0.0034 (17)
C3	0.051 (2)	0.053 (3)	0.046 (2)	0.005 (2)	−0.0033 (18)	−0.008 (2)
C4	0.056 (3)	0.044 (3)	0.061 (3)	0.002 (2)	0.008 (2)	−0.012 (2)
C5	0.064 (3)	0.041 (3)	0.064 (3)	0.001 (2)	0.023 (2)	−0.001 (2)
C6	0.057 (2)	0.044 (3)	0.044 (2)	0.001 (2)	0.0068 (19)	0.0031 (19)
C7	0.059 (3)	0.055 (3)	0.039 (2)	−0.011 (2)	0.0124 (19)	−0.0056 (19)
C8	0.050 (2)	0.055 (3)	0.042 (2)	0.006 (2)	0.0146 (18)	0.0039 (19)
C9	0.058 (3)	0.073 (4)	0.086 (4)	−0.008 (3)	0.027 (3)	−0.001 (3)
C10	0.069 (4)	0.085 (5)	0.134 (6)	−0.001 (4)	0.054 (4)	0.006 (4)
C11	0.085 (4)	0.079 (5)	0.165 (8)	0.016 (4)	0.074 (5)	−0.007 (5)
C12	0.076 (4)	0.052 (3)	0.114 (5)	−0.001 (3)	0.043 (3)	−0.012 (3)

### Geometric parameters (Å, °)

**Table:**

Co1—O1	2.150 (3)	C1—C2	1.521 (6)
Co1—O2	2.162 (3)	C2—C3	1.389 (6)
Co1—O3	2.151 (3)	C3—C4	1.365 (7)
Co1—O5	2.153 (3)	C3—H3	0.9300
Co1—N1	2.284 (4)	C4—C5	1.361 (7)
Co1—N2	2.274 (3)	C4—H4	0.9300
O1—H1A	0.8200	C5—C6	1.374 (6)
O1—H1B	0.784 (18)	C5—H5	0.9300
O2—H2A	0.8200	C6—H6	0.9300
O2—H2B	0.771 (16)	C7—C8	1.517 (6)
O3—C1	1.255 (5)	C8—C9	1.380 (7)
O4—C1	1.238 (5)	C9—C10	1.359 (8)
O5—C7	1.261 (5)	C9—H9	0.9300
O6—C7	1.222 (5)	C10—C11	1.371 (9)
N1—C8	1.321 (6)	C10—H10	0.9300
N1—C12	1.327 (6)	C11—C12	1.383 (8)
N2—C6	1.334 (5)	C11—H11	0.9300
N2—C2	1.335 (5)	C12—H12	0.9300
			
O1—Co1—O2	84.68 (13)	N2—C2—C1	116.2 (3)
O1—Co1—O3	167.36 (12)	C3—C2—C1	121.8 (4)
O1—Co1—O5	98.78 (12)	C4—C3—C2	118.2 (4)
O2—Co1—O3	92.63 (13)	C4—C3—H3	120.9
O2—Co1—O5	95.35 (13)	C2—C3—H3	120.9
O3—Co1—O5	93.75 (12)	C5—C4—C3	120.0 (4)
O1—Co1—N1	86.44 (14)	C5—C4—H4	120.0
O2—Co1—N1	163.96 (15)	C3—C4—H4	120.0
O3—Co1—N1	98.83 (14)	C4—C5—C6	119.1 (5)
O5—Co1—N1	72.84 (12)	C4—C5—H5	120.5
O1—Co1—N2	93.86 (12)	C6—C5—H5	120.5
O2—Co1—N2	98.99 (14)	N2—C6—C5	122.0 (4)
O3—Co1—N2	74.33 (12)	N2—C6—H6	119.0
O5—Co1—N2	161.68 (13)	C5—C6—H6	119.0
N1—Co1—N2	94.91 (13)	O6—C7—O5	125.9 (5)
Co1—O1—H1A	109.5	O6—C7—C8	118.7 (4)
Co1—O1—H1B	122 (3)	O5—C7—C8	115.4 (4)
H1A—O1—H1B	123.0	N1—C8—C9	122.2 (4)
Co1—O2—H2A	109.5	N1—C8—C7	116.0 (4)
Co1—O2—H2B	132 (2)	C9—C8—C7	121.9 (5)
H2A—O2—H2B	118.0	C10—C9—C8	119.5 (5)
C1—O3—Co1	119.8 (3)	C10—C9—H9	120.2
C7—O5—Co1	121.5 (3)	C8—C9—H9	120.2
C8—N1—C12	118.1 (4)	C9—C10—C11	119.0 (5)
C8—N1—Co1	114.3 (3)	C9—C10—H10	120.5
C12—N1—Co1	127.5 (3)	C11—C10—H10	120.5
C6—N2—C2	118.6 (4)	C10—C11—C12	118.1 (6)
C6—N2—Co1	128.5 (3)	C10—C11—H11	120.9
C2—N2—Co1	112.8 (3)	C12—C11—H11	120.9
O4—C1—O3	125.3 (4)	N1—C12—C11	123.0 (6)
O4—C1—C2	118.2 (4)	N1—C12—H12	118.5
O3—C1—C2	116.6 (4)	C11—C12—H12	118.5
N2—C2—C3	122.0 (4)		

### Hydrogen-bond geometry (Å, °)

**Table:**

*D*—H···*A*	*D*—H	H···*A*	*D*···*A*	*D*—H···*A*
O1—H1B···O4^i^	0.784 (18)	1.98 (3)	2.733 (4)	161 (4)
O1—H1A···O5^ii^	0.82	1.88	2.679 (4)	164
O2—H2B···O4^iii^	0.771 (16)	1.959 (16)	2.712 (4)	166 (3)
O2—H2A···O6^ii^	0.82	1.96	2.699 (5)	149

Symmetry codes: (i) *x*+1/2, −*y*+3/2, *z*+1/2; (ii) −*x*+3/2, *y*−1/2, −*z*+3/2; (iii) −*x*+1, −*y*+2, −*z*+1.
